The article "Validation of Balance Map Analysis of Walking at Different Speeds" was published in 2022. Journal: Appl Bionics Biomech.

# Validation of Balance Map Analysis of Walking at Different Speeds

**DOI:** 10.1155/2022/9268134

**Published:** 2022-03-23

**Authors:** Takahiro Kagawa

**Affiliations:** Department of Mechanical Engineering, Faculty of Engineering, Aichi Institute of Technology, 1247 Yachigusa, Yakusa-cho, Toyota 470-0392, Japan

## Abstract

Walking balance about falling in the forward direction is associated with the body's center of mass and placement of the swing foot during the swing phase. Balance map analysis evaluates walking balance based on the prediction of the reachability of an appropriate foot placement using a simple biomechanical model during the swing phase without active joint torque (ballistic walking model). The ballistic walking model can be justified in terms of the preferred walking speed because the metabolic energy consumption associated with muscle activity in faster and slower walking is higher than that in preferred speed walking. Therefore, the assumption that the active joint torque is sufficiently small during the swing phase may not hold in faster or slower walking, which can be a significant limitation of balance map analysis. In this study, it was hypothesized that steady-state walking at various walking speeds would be evaluated as stable for validation of the balance map analysis, and the gait patterns for three types of walking speeds (slow, normal, and fast) were examined. The results showed that the trajectories during the swing phase were within stable regions for all conditions, with a sufficient margin from the forward balance loss region. In addition, the margin from forward balance was reduced with an increase in walking velocity. The decrease in the margin during fast walking resulted from an increase in the forward velocity of the body's center of mass in relation to the velocity of the swing leg. These results suggest that balance map analysis effectively measures walking balance at various speeds.

## 1. Introduction

Bipedal locomotion is a fundamental motor skill of daily life. The fall risk in elderly people and people with leg motor function disabilities is higher than that in younger people without disabilities. Falls can cause serious injuries such as fractures or head injuries [1–3]. Fall-related injuries are a major cause of gait impairment, and their incidence is increasing in the aging population globally. Balance skill training can help reduce the risk [4]. For an effective intervention, a quantitative evaluation of the balance of individual walking patterns is important.

In static cases such as quiet standing, the horizontal position of the body's center of mass (COM) must be within the base of support. Expanding on the static balance stability condition, Pai and Patton proposed a dynamic stability measure as a feasible stability region in the state space of the position and velocity of the body's COM [5]. If the position and velocity of the body's COM are within the stable region, the COM of the body can be stopped within the base of the support. Otherwise, a recovery step is required to avoid falling. The extrapolated center of mass (XcoM) is a similar balance measure based on an inverted pendulum [6, 7]. The XcoM is defined as the sum of the position of the body's COM and the velocity component. If XcoM is within the base of support, the COM of the body can converge to XcoM. The feasible stability region and XcoM are effective for slip-induced backward balance losses [8] and lateral balance losses [9]. However, measures based on the inverted pendulum for the assessment of forward balance are controversial. Even if steady-state walking is maintained, these measures evaluate the state as unstable along the forward direction because the body's COM moves forward over the base of support [10]. This conflict was caused by the lack of a component of the swing leg movement in the inverted pendulum model. Walking can be stable if appropriate foot placement of the swing leg is expected before heel strike.

To deal with the contribution of the swing leg movement, we proposed a balance measure framework termed as balance map analysis [11, 12], which is based on a prediction made using a compass gait model without active joint torque (ballistic walking model [13]). When the prediction of the trajectories by the compass gait model satisfies the condition of appropriate foot placement, the state during walking is regarded as stable. Our previous study revealed that balance map analysis can detect forward balance loss when a participant is exposed to stumbling perturbation [12]. However, physiological studies raise the concern that the assumption of no active torque in the ballistic walking model may prevent its application to a wide spectrum of walking patterns. The metabolic energy consumption during walking is minimum at the preferred walking speed, and the increase in energy consumption during faster or slower walking is related to greater muscle effort than that during preferred speed walking [14]. Electromyography studies have shown that muscle activity increases with walking speed for forward propulsion [15, 16]. These studies imply that the ballistic walking concept would not be justified for faster or slower walking speeds. However, the muscle synergy analysis revealed that the muscle activities around the double support phase are mainly modulated by walking speed [17], which supports the assumption that ballistic walking can be generalized for a wide range of walking speeds.

This study is aimed at validating balance map analysis for faster and slower walking than the preferred speed. It is hypothesized that balance map analysis can evaluate steady-state walking at faster and slower speeds as stable. The stability of steady-state walking for three types of walking speeds (slow, normal, and fast) has been evaluated by balance map analysis. The similarities and differences among the conditions and validity of the balance map analysis are discussed.

## 2. Materials and Methods

### 2.1. Participants

Nine young healthy male participants participated in this experiment (age 23 ± 0.6 years, height 171.8 ± 4.2 cm, weight 61.9 ± 6.9 kg). None of the participants reported any neurological or musculoskeletal disease. The protocols for this study were approved by the ethics committee of Nagoya University. The participants explained the experiment, and they provided written informed consent before the experiment was conducted.

### 2.2. Protocol

Three conditions of walking speed (slow, normal, and fast) were tested, and the participants were instructed to walk at self-selected slow, normal, and fast speeds along a straight line on the floor. Fifteen trials were conducted for each condition. The walking distance in each trial was approximately 8 m. Before the measurement trials, participants practiced walking at each walking speed. As shown in Figure 1(a), kinematic data were collected using a three-dimensional position measurement device (Optotrak Certus, Northern Digital Inc.) at 100 Hz. Ten LED markers were attached to the heels, ankles (lateral malleoli), knees (lateral epicondyles), hips (greater trochanters), and shoulders (acromions) on both sides to evaluate the position of the COM of the body segments of the 7-link kinematics model shown in Figure 1(b). To avoid occlusion of camera markers, the participants were asked to fold their arms while walking. To acquire the time for heel strike and toe-off, pressure sensors (FSR-406, Interlink Electronics) were attached to the shoe soles, and pressure data were recorded using a 16-bit AD converter (USB-6343, National Instruments) at 100 Hz. The position and foot pressure data were simultaneously recorded using a custom software.

### 2.3. Analysis

#### 2.3.1. Balance Map Analysis

Balance map analysis is based on ballistic walking of a linear compass gait model [11, 12]. This section introduces a variable transformation to obtain the trajectory on the balance map. The compass gait model is illustrated in Figure 2. The mass point of *m*_*st*_ is the COM of the stance leg and upper body (head, arms, and trunk). Another mass point, *m*_*sw*_, is the COM of the swing leg. *l*_*st*_ is the distance between the positions of the mass point *m*_*st*_ and stance ankle joint. *l*_*sw*_ is the distance between the mass point *m*_*sw*_ and hip joint. The position of the stance leg *x*_*st*_ is defined by the horizontal position of the mass point *m*_*st*_ in relation to the stance ankle position. The position of the swing leg *x*_*sw*_ is defined as the horizontal position of the distal point of a line segment from the hip position via the mass point *m*_*sw*_ with a length of *l*_*st*_.

The linearized equation of motion for the compass gait model is represented by the following equation:

(1) $$\begin{array}{c} \left(\begin{array}{c} {\ddot{x}}_{st}\\ {\ddot{x}}_{sw} \end{array}\right)=\left(\begin{array}{cc} \frac{\Omega_{st}^{2}}{K} & \frac{\left(1-K\right)\Omega_{st}^{2}}{K}\\ -\frac{\Omega_{sw}^{2}}{K} & -\frac{\Omega_{sw}^{2}}{K} \end{array}\right)\left(\begin{array}{c} x_{st}\\ x_{sw} \end{array}\right), \end{array}$$

where $\Omega_{st}=\sqrt{l_{st}/g}$, $\Omega_{sw}=\sqrt{l_{sw}/g}$, and *K* = *m*_*st*_/(*m*_*st*_ + *m*_*sw*_). Balance map analysis determined that the states $\left(x_{st},x_{sw},{\dot{x}}_{st},{\dot{x}}_{sw}\right)$ are stable if the ballistic trajectories *x*_*st*_(*t*) and *x*_*sw*_(*t*) of the state intersect at least once during the late swing phase (x_*sw*_ > 0). In steady-state human walking, the posture at heel strike in the sagittal plane is symmetrical [18], which corresponds to the intersection of the trajectory (*x*_*st*_ = *x*_*sw*_). Therefore, the existence of an intersection means that an appropriate foot placement is reachable to continue steady-state walking.

To simplify the analytical solution of Equation (1), two variable transformations were introduced. The first variable transformation decouples the stance and swing leg positions, which are given by:

(2) $$\begin{array}{c} \left(\begin{array}{c} {\hat{x}}_{st}\\ {\hat{x}}_{sw} \end{array}\right)=\left(\begin{array}{cc} \Omega_{st}^{2} & K\omega_{sw}^{2}\\ \Omega_{st}^{2} & -K\omega_{st}^{2} \end{array}\right)\left(\begin{array}{c} x_{st}\\ x_{sw} \end{array}\right), \end{array}$$

where

(3) $$\begin{array}{c} \omega_{st}^{2}=\Delta \Omega +\sqrt{\Delta \Omega^{2}+4K\Omega_{st}^{2}\Omega_{sw}^{2}},\\ \omega_{sw}^{2}=-\Delta \Omega +\sqrt{\Delta \Omega^{2}+4K\Omega_{st}^{2}\Omega_{sw}^{2}},\\ \Delta \Omega =\Omega_{st}^{2}-\Omega_{sw}^{2}. \end{array}$$

When *x*_*st*_ = *x*_*sw*_, the transformed variables ${\hat{x}}_{st}$ and ${\hat{x}}_{sw}\;$ satisfy ${\hat{x}}_{st}=x_{st}$ and ${\hat{x}}_{sw}=x_{sw}$. The analytical solutions of the stance and swing leg positions follow:

(4) $$\begin{array}{c} {\hat{x}}_{st}\left(t\right)=\left\{\begin{array}{cc} \frac{\sqrt{2E_{st}}}{\omega_{st}}\sinh\left(\omega_{st}t+\psi_{st}\right) & \text{for }E_{st}>0\\ \pm \frac{\sqrt{2E_{st}}}{\omega_{st}}\cosh\left(\omega_{st}t+\psi_{st}\right) & \text{for }E_{st}<0 \end{array}\right., \end{array}$$

(5) $$\begin{array}{c} {\hat{x}}_{sw}\left(t\right)=\frac{\sqrt{2E_{sw}}}{\omega_{sw}}\sin\left(\omega_{sw}t+\psi_{sw}\right). \end{array}$$

*E*_*st*_ and *E*_*sw*_ represent energy exhibited by

(6) $$\begin{array}{c} E_{st}=\frac{1}{2}{\left(\frac{d{\overset{\wedge }{x}}_{st}}{dt}\right)}^{2}-\frac{1}{2}{\left(\omega_{st}{\overset{\wedge }{x}}_{st}\right)}^{2}, \end{array}$$

(7) $$\begin{array}{c} E_{sw}=\frac{1}{2}{\left(\frac{d{\overset{\wedge }{x}}_{sw}}{dt}\right)}^{2}+\frac{1}{2}{\left(\omega_{sw}{\overset{\wedge }{x}}_{sw}\right)}^{2}. \end{array}$$

*ψ*_*st*_ and *ψ*_*sw*_ are the phases of each function provided by

(8) $$\begin{array}{c} \psi_{st}\left(t\right)=\left\{\begin{array}{cc} \tanh^{-1}\left\{\frac{\omega_{st}{\hat{x}}_{st}}{{\dot{\hat{x}}}_{st}}\right\} & \text{for }E_{st}>0\\ \tanh^{-1}\left\{\frac{{\dot{\hat{x}}}_{st}}{\omega_{st}{\hat{x}}_{st}}\right\} & \text{for }E_{st}<0 \end{array}\right., \end{array}$$

(9) $$\begin{array}{c} \psi_{sw}\left(t\right)=\tan^{-1}\left\{\frac{\omega_{sw}{\hat{x}}_{sw}}{{\dot{\hat{x}}}_{sw}}\right\}. \end{array}$$

The parameter values of the energy and phase were constant for the ballistic trajectories of the stance and swing leg positions.

To simplify solutions (4) and (5), the second variable transformation of nondimensionalization for position *χ* and time *T* is introduced:

(10) $$\begin{array}{c} \chi =\frac{\omega_{sw}}{\sqrt{2E_{sw}}}\hat{x,}T=\omega_{sw}t+\psi_{sw}. \end{array}$$

The trajectories of nondimensional position solutions *χ*_*st*_(*T*) and *χ*_*sw*_(*T*) are represented by

(11) $$\begin{array}{c} \chi_{st}\left(T\right)=\left\{\begin{array}{cc} \frac{\sqrt{E_{n}}}{\omega_{n}}\sinh\left(\omega_{n}T+\psi_{n}\right) & \text{for }E_{n}>0\\ \pm \frac{\sqrt{-E_{n}}}{\omega_{n}}\cosh\left(\omega_{n}T+\psi_{n}\right) & \text{for }E_{n}<0 \end{array}\right., \end{array}$$

(12) $$\begin{array}{c} \chi_{sw}\left(T\right)=\sin T. \end{array}$$

Equations (11) and (12) imply that the relationship between the stance and swing trajectories can be determined based on three parameters: the natural frequency ratio *ω*_*n*_ = *ω*_*st*_/*ω*_*sw*_, energy ratio *E*_*n*_ = *E*_*st*_/*E*_*sw*_, and phase difference *ψ*_*n*_ = *ψ*_*st*_ − *ω*_*n*_*ψ*_*sw*_. The natural frequency ratio *ω*_*n*_ is related to human anthropometric parameters (e.g., *m*_*st*_, *m*_*sw*_, *l*_*st*_, and *l*_*sw*_), and the energy ratio and phase difference are determined by the current state $\;\left(x_{st},x_{sw},{\dot{x}}_{st},{\dot{x}}_{sw}\right)$. The energy ratio represents the forward movement ability of the stance leg position relative to the swing leg position. If *E*_*n*_ < 0, the stance leg position cannot move forward, which corresponds to backward balance loss [19]. If *E*_*n*_ ≫ 1, the velocity of the stance leg is much faster than the swing leg, and the state is close to falling forward. The phase difference represents the position of the stance leg relative to that of the swing leg. The delay in the phase difference (*ψ*_*n*_ < 0) indicates that the stance leg is located posterior to the swing leg, and there is a large margin for forward falling. The advance of the phase difference (*ψ*_*n*_ > 0) indicates the anterior location of the stance leg position and a lower margin for forward fall. As the energy ratio and phase difference are deterministic parameters of ballistic trajectories, there are upper and lower boundaries of the parameter sets that the trajectory of the stance leg position intersects that of the swing leg position. The upper and lower boundaries of the parameter sets were calculated using a binary-search algorithm.

To represent the balance state intuitively, the balance map shown in Figure 3 depicts the regions in which the ballistic trajectory from the current state has an intersection (stable touchdown) or not (balance loss) in the state space at = 0$\left(\chi_{st0},{\dot{\chi }}_{st0}\right)$, where *χ*_*sw*_ = 0 at *T* = 0. The dashed curves and radial lines are contour plots of the energy ratio and phase difference, respectively. The location on the balance map was determined by a set of energy ratios and phase differences. The state in the stable touchdown region (unfilled region) indicates that at least one intersection exists between the stance and swing trajectories. When the state is in the forward balance loss region, there is no intersection between trajectories. The state in the backward balance loss region (*E*_*n*_ <0 and *χ*_*st*0_ < 0) indicated that the trajectory of the stance leg could not move forward across the stance ankle position without energy input.

#### 2.3.2. Data Processing

The measured kinematic data were low-pass filtered using an FIR filter with a cut-off frequency of 10 Hz. The marker positions of the ankles, knees, and hips were regarded as the center of joint rotation of the 7-link model in the sagittal plane (Figure 1(b)). The proximal joint position, angle about the horizontal axis, and length of each body segment were calculated using the kinematic data. The COM positions of the body segments were calculated based on typical anthropometric parameters (segment weight/body weight and the segment center of mass/segment length) derived by [20]. The time at toe-off and heel strike was determined using foot pressure data. The data from the first and last two cycles, each, were removed from the analysis to evaluate steady-state walking [21]. The period of each walking cycle was calculated as the duration between two consecutive heel strikes. The stride length of each cycle was evaluated based on the distance between the heel positions of two consecutive heel strikes. The walking velocity in each cycle was calculated by dividing the stride length by the period.

Based on the preprocessed kinematic data, the position and velocity of the stance and swing legs $\left(x_{st}\left(t_{i}\right),x_{sw}\left(t_{i}\right),{\dot{x}}_{st}\left(t_{i}\right),{\dot{x}}_{sw}\left(t_{i}\right)\right)$ during the swing phase were calculated. Although balance map analysis assumes that the stance leg position is regarded as the position of the hip joint, there is an error between the stance leg and horizontal hip joint positions. The average absolute error was 0.01 m which is approximately 2% of the movement distance during a step. Applying the variable transformation of Equation (2) for decoupling, the parameter values of the energy ratio *E*_*n*_(*t*_*i*_) and phase difference *ψ*_*n*_(*t*_*i*_) were calculated based on Equations (6)–(9). Substituting *E*_*n*_(*t*_*i*_), *ψ*_*n*_(*t*_*i*_), and *T* = 0 into Equation (11) and its derivative, the state on the balance map ($\chi_{st0}\left(t_{i}\right),{\dot{\chi }}_{st0}\left(t_{i}\right)$) was obtained. Walking balance can be quantified by the margin between the state ($\chi_{st0}\left(t_{i}\right),{\dot{\chi }}_{st0}\left(t_{i}\right)$) and nearest neighbor point on the boundary of the balance loss region $\left(\bar{\chi },\bar{\dot{\chi }}\right)$ as follows:

(13) $$\begin{array}{c} D\left(t_{i}\right)=\sqrt{{\left({\dot{\chi }}_{st0}\left(t_{i}\right)-\bar{\dot{\chi }}\right)}^{2}+\omega_{n}^{2}{\left(\chi_{st0}\left(t_{i}\right)-\bar{\chi }\right)}^{2}}. \end{array}$$

#### 2.3.3. Statistical Analysis

The differences in the spatio-temporal parameters (velocity, stride, and period) among conditions (slow, normal, and fast) were statistically tested using repeated measure analysis of variance (ANOVA). The average trajectory on the balance map of each condition and each participant was calculated by averaging the time-normalized trajectories by cubic interpolation. The difference in the margin with two factors of walking speed (slow, normal, and fast) and the phase (initial, mid-, and terminal swing) was examined using two-way repeated measures ANOVA. The initial and terminal swing phases were defined by the timing of the toe-off and heel strike, respectively. The midswing phase is the intermediate time between toe-off and heel strike. The normality assumption of the data distribution was examined using the Jarque-Bella test, and the sphericity of covariance was tested using Mauchly's test. If the sphericity assumption was violated, the Greenhouse-Geisser correction was adopted. The post hoc test of the paired *t*-test with Bonferroni correction was performed to determine the differences among the conditions. In addition to the significance based on the *p* value, the effect sizes of ANOVAs (partial eta squared) and post hoc paired *t*-tests (Cohen's *d*) were evaluated. Changes in the energy ratio and phase difference related to walking velocity were evaluated using regression analysis. The significance level for all statistical tests was set at 5%. Statistical tests were performed using the Statistics and Machine Learning Toolbox of MATLAB 2019a (MathWorks, Inc.).

## 3. Results

The average and SD of the walking speed, stride length, and period for each walking speed condition are listed in Table 1. The velocity among all conditions and participants ranged from 0.6 to 1.7 m/s while the average normal speed was less than the standard average value (1.2–1.4 m/s) [22]. The normality tests of the distributions of walking speed, stride length, and periods in each condition did not show a significant deviation from normality. ANOVA showed that the differences in walking speed were significant among the conditions (*F* (1.09, 8.71) = 120.81, *p* < 0.01, *η*_*p*_^2^ = 0.94). Stride length and period were also significantly different between the conditions (stride length: *F* (2, 16) = 117.04, *p* < 0.01, *η*_*p*_^2^ = 0.93, period: *F* (1.05, 8.42) = 54.31, *p* < 0.01, *η*_*p*_^2^ = 0.87). The post hoc tests revealed that the parameters of each condition were significantly different from those of the other conditions (Table 2). The stride length increased, and the period of the gait cycle decreased with gait velocity.

Figure 4 shows the average trajectories on the balance map under slow, normal, and fast conditions for a typical participant. The trajectories were within the stable touchdown region, and their shapes were similar. The trajectories of all participants exhibited similar properties.  Figure 5 shows the margin from the boundary line of the forward balance loss region at the initial, mid-, and terminal swing phases for all participants. The results of the normality tests of the distributions of the margin at each condition were not significant, except for the slow condition at the initial swing phase. ANOVA revealed significant effects of walking speed (*F* (1.14, 9.20) = 27.4, *p* < 0.05, *η*_*p*_^2^ = 0.77) and phase (*F* (1.51, 12.09) = 267.3, *p* < 0.05, *η*_*p*_^2^ = 0.97) and a significant interaction (*F* (2.52, 20.16) = 10.80, *p* < 0.05, *η*_*p*_^2^ = 0.57). The results of the post hoc tests are summarized in Table 3. There were significant differences among all combinations of walking speeds during the initial and midswing phases. In the terminal swing phase, a significant difference was found between the normal and fast phases. Statistical analysis revealed that the margin from the forward balance loss region decreased with an increase in walking speed.

Figure 6(a) shows the results of the regression analysis of walking velocity and energy ratio. The energy ratio increased with the velocity, and the regression was significant (*R*^2^ = 0.48, *p* < 0.05).  Figure 6(b) shows the results of the regression analysis of walking velocity and phase difference. The phase difference was almost constant among the conditions, and the regression was not significant (*R*^2^ = 0.12, *p* = 0.08). The phase difference was negative (−0.12), which was beneficial for enlarging the margin of forward balance loss.

## 4. Discussion

In this study, the experimental results exhibited both similarities and differences in trajectories during steady-state walking on a balance map considering different walking speed conditions. The major finding of this study was that the trajectories on the balance map were within the stable touchdown region under slow, normal, and fast walking conditions. The assumption of ballistic walking concerns the prediction error in slower and faster walking, owing to greater metabolic costs and muscle activity. However, the measured trajectories under slow and fast walking conditions were within the stable touchdown region and exhibited a shape similar to the trajectory of the normal walking condition (Figure 4). The margin from the forward balance loss indicated that the trajectories of all the participants were within the stable touchdown region with sufficient margins (Figure 5). The average of the preferred walking speed in this experiment (1.07 m/s) was less than the standard preferred walking speed (around 1.2–1.4 m/s) [22]. One of the possible reasons for the slower speed was the short walking path (8 m). However, steady-state gait data ranging from 0.6 to 1.7 m/s satisfied the stable touchdown condition. Therefore, we conclude that balance map analysis can be applied to gait kinematics data for a wide range of walking speeds. A previous study reported increased muscle activity with walking speed, while a speed-dependent change in muscle activity was found in the late stance phase and early swing phase for push-off [17]. In addition, Neptune et al. [23] reported that the increased positive work of the muscles with velocity during the swing phase was smaller than that during the stance phase. Our conclusion does not contradict these physiological and biomechanical studies.

The second finding was that the margin from the forward balance loss on the balance map depended on the walking speed from the early to the middle of the swing phase. A higher walking speed resulted in a smaller margin of forward balance loss (Figure 5). This is consistent with the results of the data-driven approach proposed by Pavol et al. [24]. Pavol et al. reported horizontal hip velocity as the greatest cause of falling after tripping in healthy older adults. In our study, the decrease in the margin resulted from an increase in the energy ratio, rather than an increase in the phase difference because the energy ratio was significantly correlated with the walking velocity (Figure 6(a)). A higher energy ratio indicates faster horizontal movement of the body's COM relative to the velocity of the swing leg position. On the other hand, the phase differences were delayed for all walking speed conditions (Figure 6(b)). The delay of the phase difference indicates that the swing leg position is anterior to the stance leg position (i.e., the COM position of the horizontal body), which improves the likelihood of enabling appropriate foot placement before falling. In the future, we will investigate the mechanism of the increase in forward fall risk with walking velocity from a biomechanical perspective.

The measures of walking balance based on the inverted pendulum model are well established for backward and lateral balance loss [5–7]. Based on the extrapolated COM concept, one may fall backward if the position of the XcoM is located posterior to the base of the support during walking. On the other hand, if the XcoM is located anterior to the base of the support during walking, one may not fall forward immediately. The swing foot lands on the floor before falling and generates the next base of support. The XcoM located much anterior to the base of support may indicate that the body's COM is too fast for appropriate placement of the swing leg [25]. However, it is difficult to determine a clear threshold of XcoM to detect forward balance loss in steady-state walking because the inverted pendulum model does not involve swing leg movement. Balance map analysis defines the forward balance loss by the reachability of the stable touchdown condition predicted by an analytical solution of the linear compass gait model. A clear measure of forward and backward balance loss is beneficial for assessing fall risk during walking.

One of the limitations of this study is the simplicity of the measurement setup and kinematics model of human gait. The gait pattern was measured using ten markers, and the head, arms, and trunk were regarded as a rigid body in the 7-link kinematics model. This simplification was based on the assumption that an upright posture of the upper body was maintained during walking of normal people. However, the simple maker placement and kinematics model would be problematic for evaluating abnormal gait patterns. Measurement with more markers and a detailed kinematics model would be required to evaluate abnormal gait patterns because complex movements of the upper body are one of the common properties of abnormal gait. Another limitation is the low walking velocity of the measured gait patterns. It is supposed that the participants selected slower walking velocity than usual because of the short walking path in the experiment setup. In addition, it is still unclear whether the balance map analysis is feasible for walking with maximum velocity (transition velocity from walk to run). Further investigation is needed to specify the feasible range of walking velocity for the balance map analysis.

## 5. Conclusion

It was confirmed that balance map analysis can evaluate the walking stability of steady-state walking at different walking speeds. In addition, the margin for forward falling reduced with an increase in walking velocity, which is consistent with previous data-driven studies. The smaller margin was caused by the high horizontal velocity of the body's COM relative to the horizontal velocity of the swing leg.

## Figures and Tables

**Figure 1:** Measurement of human gait and analysis of gait kinematics for calculation of the COM of the body segments. (a) Measurement of the positions of the heel, ankle, knee, hip, and shoulder joints of the left and right sides by a motion capture system (OPTOTRAK). (b) The COM of the feet, shanks, thighs, and head-arms-trunk segments were estimated by a 7-link kinematics model.

**Figure 2:** Two-link model (compass gait model) with the stance leg and swing leg.

**Figure 3:** Stable touchdown (unfilled region) and balance loss regions (filled regions) in the state space of nondimensional stance leg position, which is referred to as the balance map. The filled region in *E*_*n*_ < 0 and *χ*_*st*_ < 0 is the backward balance loss region. Another filled region is the forward balance loss region.

**Figure 4:** Average trajectories on the balance map under slow (a), normal (b), and fast (c) walking conditions for a typical participant. The blue, green, and red ellipses are 95% confidence ellipses at the initial swing, midswing, and terminal swing phases, respectively.

**Figure 5:** Margin from the forward balance loss of each participant at initial swing (a), midswing (b), and terminal swing (c).

**Figure 6:** Results of regression analyses between the walking velocity and energy ratio (a) and between the walking velocity and phase difference (b). The dashed line in each figure corresponds to the mean value under all the conditions (${\bar{E}}_{n}=0.22$, ${\bar{\psi }}_{n}=-0.12$).

**Table 1:** Average and standard deviation of the gait parameters (velocity, stride length, and period) of measured walking data.

	Slow	Normal	Fast
Velocity, m/s	0.72 (0.10)	1.07 (0.09)	1.44 (0.14)
Stride length, m	1.06 (0.11)	1.26 (0.08)	1.45 (0.09)
Period, s	1.48 (0.16)	1.17 (0.08)	1.01 (0.08)

**Table 2:** Statistical results of post hoc test of walking speed.

	Velocity		Stride		Period	
	*p* value	Cohen's *d*	*p* value	Cohen's *d*	*p* value	Cohen's *d*
Slow vs. normal	*p* < 0.01	3.21	*p* < 0.01	2.34	*p* < 0.01	2.21
Slow vs. fast	*p* < 0.01	3.75	*p* < 0.01	4.33	*p* < 0.01	2.54
Normal vs. fast	*p* < 0.01	3.88	*p* < 0.01	4.01	*p* < 0.01	2.89

**Table 3:** Statistical results of post hoc test of margin among the conditions of walking speed by phase.

	Initial swing		Midswing		Terminal swing	
	*p* value	Cohen's *d*	*p* value	Cohen's *d*	*p* value	Cohen's *d*
Slow vs. normal	*p* < 0.01	1.37	*p* < 0.05	1.26	*p* = 0.27	0.63
Slow vs. fast	*p* < 0.01	1.75	*p* < 0.01	1.77	*p* = 0.06	0.98
Normal vs. fast	*p* < 0.01	1.28	*p* < 0.01	2.14	*p* < 0.05	1.29

## Data Availability

The data and code used in this study are available from the corresponding author upon request.
